The article "Effect of Nursing Intervention on Coronary CT Angiography in Elderly Patients" was retracted in 2023. Reasons: unreliable results or conclusions; lack of ethics approval or compliance; concerns about the data; concerns about the peer review.

# Effect of Nursing Intervention on Coronary CT Angiography in Elderly Patients

**DOI:** 10.1155/2022/3663285

**Published:** 2022-06-16

**Authors:** Yajuan Yin, Zhongting Wei

**Affiliations:** ^1^School of Nursing Science, Guangxi University of Science and Technology, Liuzhou, Guangxi 545006, China; ^2^Guangxi University of Science and Technology Second Hospital, Liuzhou, Guangxi 545006, China

## Abstract

To investigate the clinical benefits of coronary CT angiography in older adults. The results of this trial were 110 patients who underwent CT angiography (selected from 20 March 2016 to 20 March 2017). Use computer group mode. The control group received health care, including 50 patients, and the control group received usual care, including 60 patients. Then, the best and best image quality, time-consuming analysis, and satisfaction were compared between the two groups. The experimental results showed that the best and best image quality (83.00%), examination time (5.72 ± 1.81) minutes, and patient satisfaction (100.00%) of the experimental group were better than those of the control group (*P* < 0.05). Targeted healthcare for patients undergoing coronary CT angiography can improve the patient's ability to receive a diagnosis with a consistent attitude, reduce work hours, reduce adverse factors, and improve patient satisfaction with care.

## 1. Introduction

Coronary heart disease is a fatal heart disease that kills many people. The literature shows that heart disease accounts for about 15% of all deaths and has a significant impact on the life and health of patients [1]. Early diagnosis and early treatment are important ways to reduce cardiovascular mortality and improve prognosis. Conventional coronary angiography (CAG) is the gold standard for diagnosing coronary heart disease, but treatment is limited by high costs. CT coronary angiography (CTCA) is widely used for the diagnosis of coronary heart disease because of the physical improvement and resolution of a large number of CT films. However, how to reduce patient discomfort, complete screening, and good imaging has become an important part of electrical research [2]. Multislice spiral CT coronary angiography (MSCTCA) is a new, concealed, and safe device that has been widely used in hospitals. MSCTCA can be used as a first-line diagnosis and clinical examination of vascular stenosis. The sensitivity, specificity, and accuracy of its measurements have been recognized, leading to better and more accurate treatments for hospitals [3].

Coronary CT angiography (Figure 1) is an important basis for screening and preliminary diagnosis of coronary intervention at present. It belongs to a new diagnostic mode. It has the advantages of safety, noninvasive, high-diagnostic accuracy, and simple operation. It has high sensitivity and specificity for coronary artery and can accurately evaluate the degree of lesions, so as to provide basis for the formulation of treatment plan. However, with the deepening of relevant reports, it can be found that the CT angiography of coronary artery can be affected by factors such as environment, psychology, respiratory coordination, and heart rate. In this regard, it is also necessary to strengthen nursing intervention and guidance, so as to ensure image quality and improve the success rate of examination. Routine nursing is more passive and one-sided, which is not conducive to wide promotion. Therefore, targeted nursing intervention should be selected to improve the imaging quality by standardizing the nursing before, during, and after the examination. This paper is aimed at exploring the value of different nursing methods in patients undergoing coronary CT angiography, as described below [4].

## 2. Literature Review

Liu and others think that coronary heart disease is the abbreviation of coronary heart disease, and it is often found in the middle and old age population. With the increase of age, the incidence rate of disease is gradually increasing. CAG is the gold standard for judging the degree of coronary artery stenosis, but the examination price is high and invasive, causing serious damage to the patient's body [5]. Smeets and others believe that CTCA is a new noninvasive and safe technology with high sensitivity and specificity. How to maintain the best state of patients during examination and improve the imaging quality of CTCA has become the most concerned issue of Radiology Department [6]. Faan and others believe that CTCA is an important screening method for evaluating coronary artery disease in patients with coronary heart disease. 64 slice spiral CT has the characteristics of fast scanning, high image quality, and high diagnostic accuracy, but good nursing cooperation is an important part of successful examination, especially heart rate and psychological regulation [7]. Yang and others found that the change of heart rate plays an important role in the imaging quality of CTCA. When the heart rate is slow, CTCA can get the best imaging quality. Therefore, a stable heart rate should be maintained during the examination [8]. Msosa and others believe that the factors affecting heart rate include basic heart rate, mood fluctuation, and severity of disease. Before the examination, nurses actively communicate with patients, listen to their voices, find the source of patients' anxiety factors, explain the pathogenesis of coronary heart disease and the importance of CTCA examination through professional knowledge, patiently answer patients' questions, improve patients' understanding of CTCA examination of coronary heart disease, alleviate patients' tension, enhance their self-confidence to overcome the disease, reduce patients' psychological burden, and stabilize their heart rate [9]. Zima and others since the wide application of multislice spiral CT, the CT scanning speed have been significantly improved. The imaging mode has entered the era of three-dimensional volume scanning from two-dimensional image acquisition. Moreover, the postprocessing methods of multislice spiral CT images are diverse, which increases the application range of spiral CT [10]. Sole and others believe that CT angiography (CTA) refers to rapid spiral CT scanning while rapidly injecting contrast agent into vein, and the obtained data is processed by advanced computer to form the image of blood vessel. Cti1 examination has the advantages of small trauma, rapid examination, convenient imaging, and accurate diagnosis. This imaging examination method provides a reliable anatomical basis for surgical operation planning and plays an extremely important role in the evaluation of blood vessels before and after liver operation [11]. Alperovitch-Najenson and others believe that powerful CT postprocessing function, after scanning, dual source CT can automatically select the best phase of coronary artery development for reconstruction through prospective ECG gating equipment. When the automatic selection is wrong, manual reconstruction can also be further selected [12].

## 3. Experimental Analysis

### 3.1. Subjects

A total of 100 subjects were accepted from March 20, 2016, to March 20, 2017. The researchers divided the patients who underwent CT angiography into two groups of 40 before and after admission. The procedure includes (1) when the patient is resting, the heart rate is less than 100 beats per minute, and the breath is less than 30; (2) after the ECG examination, the patient can see the clear vision of the nasal cavity, as well as the sound quality; (3) all patients have coronary artery CT angiography indications; (4) all patients have signed the written consent [13].

Exclusion procedure: (1) exclude patients with severe arrhythmia; (2) exclude patients with congestive heart failure; (3) exclude patients with liver and kidney insufficiency and hyperthyroidism; (4) exclude patients who are allergic to iodine concentration. The mean age of the research group was (52.86 ± 3.22) years, including 26 males and 24 females [14].

### 3.2. Experimental Method

Scanning method: the CT scanner used this time adopts the light speed 61 row model provided by GE company to assist the patient in the supine position, and 350 mg/ml iohexol is injected through elbow vein. The coronary artery and intracardiac and extracardiac structures of the observation group are observed, and the patient images are processed after surface reconstruction, multiplanar reconstruction, volume reproduction, and maximum density projection. The control group was given routine nursing guidance and informed of relevant knowledge and precautions before the examination [15]. The observation group adopted targeted nursing intervention, mainly including

1. *Nursing before Examination*. ① Psychological nursing: in order to reduce the image artifacts caused by arrhythmia or rapid heart rate and maintain a stable heart rate, it is also necessary to do a good job of psychological counseling to help patients eliminate their inner tension and patiently explain the function, purpose, and relevant matters of concern of this examination. In order to prevent accidents, it is also necessary to ask the patients whether they have organ diseases and drug allergy history before examination; ① in order to ensure the accurate and smooth pushing of the contrast medium, it is also necessary to select the blood vessel puncture without puncture, phlebitis, and thick and straight on the same day and select the corresponding needle model according to the injection flow rate and blood vessel conditions. At the same time, the venous trocar has unique elasticity and flexibility, safe and simple operation, little stimulation to blood vessels, and will not lead to leakage or trocar prolapse due to high pressure or too fast injection speed [16]. After successful puncture, 1 ml of contrast medium needs to be injected and observed for 15 minutes. The examination can be continued only after it is confirmed that there is no allergic reaction; ① respiratory training: respiratory artifact is the main factor leading to the failure of the examination. For this, it is also necessary to teach the patients the correct nursing methods before the examination and reasonably adjust the respiratory rate according to the instructions of the CT machine, so as to improve the image quality. During the examination, the respiratory rate should be kept in a uniform state, the chest and abdominal wall should not move up and down, and the lips should be closed tightly. Breathe only after hearing the breath holding display light goes out or the instructions, and the breath holding time should not be pushed back. Train several times according to the method until the patients fully master and understand it. For patients with poor hypoxia tolerance or lung diseases, oxygen inhalation intervention is also needed to maintain body braking, and the patients are instructed not to sneeze, swallow, cough, and other actions; ① therefore, it is also necessary to take *β* receptor blocker before the examination, so as to control the heart rate, and so as to avoid arrhythmia and artifacts. Before the examination, ask the patient to lie down and rest for 15 minutes, and then continue the examination after the mood fluctuation is stable [17]
2. In order to avoid the failure of breath holding, breath holding training should be carried out again, and the smoothness of the indwelling needle should be checked. When injecting contrast agent, maintain the speed of 5 ml per second. In the process of examination, once the patient has abnormal phenomena, it is necessary to stop the examination immediately and give corresponding symptom intervention [18]
3. *Postexamination Care*. After the scanning is completed, separate the puncture needle and high-pressure syringe, and keep the needle for observation for 30 minutes. After the patient has no abnormalities, it can be removed. For patients with vomiting symptoms, they need to be treated with corresponding antiemetic drugs and encourage patients to drink more water to promote the discharge of contrast agent

### 3.3. Observation Indicators

The nursing satisfaction of patients was evaluated by nursing evaluation scale. The total score was 100, 80~100 was very satisfied, 60~79 was satisfied, and <59 was dissatisfied. The nursing satisfaction was (very satisfied + satisfied)/total person × 100%. Excellent rate of image quality: excellent rate = excellent rate + good rate; excellent: the vessel contour is clear, and there is no artifact in the coronary artery; good: the contour of local blood vessels is blurred or there are artifacts in local coronary arteries; poor: vessel contour is blurred or vessel display is interrupted, and artifacts appear in all or most of the coronary arteries.

### 3.4. Statistical Treatment

The statistical software SPSS 22.0 was used for data processing. The inspection time was represented by (*x* ± *s*), and the *t*-test was used; the excellent rate of image quality and nursing satisfaction of counting data are expressed in (%), and *x*^2^ test is adopted. If the final comparison result shows that *P* < 0.05, it indicates that the data difference is statistically significant [19].

### 3.5. Result Analysis

The image quality of the control group was higher than that of the control group, and the difference was statistically significant (*P* < 0.05), as shown in Table 1.

The nursing rate in the control group was higher than that in the control group, and the monitoring period was shorter than that in the control group (*P* < 0.05), as shown in Table 2.

The comparison of baseline heart rate and postoperative heart rate after the health study between the two groups is shown in Table 3. As can be seen from Table 3, there was no difference in heart rate between the two groups; after a healthy workout (waiting for a 15-minute rest), heart rate increased faster than heart rate in both groups. Compared with the group, the difference was statistically significant; after the health study, the heart rate of the control group was faster than that of the affected group. There were significant differences between the two groups.

The comparison of cardiac control time and breathing time in the combined breathing group between the two groups is shown in Table 4. As can be seen from Table 4, after oral administration of metoprolol hydrochloride, the heart rate was below 70 BPM and the time it took for the joint to breathe. Training time in both groups was shorter in the group intervention than in the control group. The difference between the two groups was significant [20].

The incidence and efficacy of heart rate > 10 bpm between the two groups are shown in Figure 2. As can be seen from Figure 2, the effect of the heart rate change > 10 bpm control group was lower than that of the control group, and the success rate was higher than that of the control group. Differences between the two groups were significantly identified.

## 4. Discussion

It can be seen from the experiment that the heart rate of the examiners in both the intervention group and the control group is faster than the basic heart rate after entering the waiting room and resting quietly for 15 minutes, which is related to the examiners' tension in the specific environment of the hospital, fear of the examination process, and strangeness to the medical staff [21]. Nervous and fearful emotions can cause the examiner's sympathetic nerve to be excited and his heart rate to increase. The faster heart rate coronary angiography, in addition to the higher chance of image artifacts, the time of image postprocessing is also significantly prolonged. Therefore, the examiner's emotional tension will increase the examiner's dose of heart rate control and prolong the time of heart rate control, resulting in the prolongation of the workflow. Its center rate is an important factor that directly affects the image quality. At present, some studies believe that when the heart rate of patients is ≤65 BPM during coronary artery imaging, relatively good image quality can be obtained. Some scholars also observed that the greater the fluctuation range of heart rate during the examination, the more obvious the decline of image quality, especially when the fluctuation range of heart rate is ≥0.5 bpm. Therefore, we routinely require that the examiner's heart rate be controlled below 70 BPM before examination. When the heart rate fluctuation amplitude is 10 bpm during the examination, it has little impact on the quality of coronary artery imaging. Some authors suggest using a receptor blocker to control heart rate. When the subject is in the routine examination room, it may be related to the increase of heart rate fluctuation when we are in the examination room or lying in the examination room. When the subject is nervous, it may be found that the heart rate of some subjects will increase when we are lying in the examination room. Some subjects need to wait for *β* long time after taking metoprolol orally for many times, and the heart rate is still difficult to control, resulting in failure of examination and prolongation of workflow, resulting in waste of personnel and equipment resources [22].

It can be seen from the experimental data that there was no significant difference in the basal heart rate between the two groups of examiners. After 15 minutes of rest in the waiting room, the heart rate in the control group was significantly higher than that in the intervention group (*P* < 0.001), and the difference was statistically significant. By fully communicating with the inspectors in the intervention group before the inspection, the inspectors have a full understanding of the entire inspection process, actively cooperate with the inspection, and reduce tension and fear [23]. At the same time, combined with oral metoprolol hydrochloride, it can quickly control the examiner's heart rate and reduce the fluctuation range of heart rate during the examination. The results showed that the heart rate control time of the examiners in the intervention group was significantly shorter than that in the control group, the incidence of heart rate fluctuations > 10 bpm during the inspection process was significantly lower than that in the control group, and the inspection success rate was significantly higher than that in the control group. It shows that effective health education and psychological nursing measures can ensure the success rate of examination while optimizing the workflow.

In the process of coronary artery imaging, it is generally necessary for the subject to hold his breath for 5 ~ 10 s, but some subjects cannot hold their breath due to tension and other reasons, resulting in respiratory motion artifacts. In order to reduce the impact of breathing on coronary artery imaging, train the examiner to hold his breath after inhaling evenly and repeat it many times until the examiner can successfully complete the inhaling and holding action within the estimated scanning time after hearing the instruction. In addition, the respiratory movement of some examiners is uneven, resulting in the selection of trigger points sometimes low and resulting in shear artifacts. Therefore, it is necessary to emphasize the importance of uniform breathing to the examiners [24]. In the control group, the technician only instructed the examiner to follow the instructions of the machine, inhale deeply first, and then hold his breath, but the examiner often breathed involuntarily, so that the technician needed to repeatedly train the examiner's breathing cooperation. In the intervention group, the nurses trained the examiners to inhale evenly before the examination and then hold their nose while holding their breath. This has a better effect, controlling the examiners' involuntary spontaneous breathing and reducing the generation of respiratory artifacts.

Coronary CTA examination should obtain excellent images. As a nursing staff, every patient can achieve the best state before the examination. Let patients actively cooperate during the examination and actively communicate with patients after the examination, which is not only to ensure clear image quality but also the main purpose of nursing work.

In terms of psychological nursing, targeted psychological intervention should be implemented before the examination to overcome the tension of patients, such as eliminating the fear of large-scale instrument examination, the harm of ionizing radiation to the body and the safety of contrast agent, so as to reduce the psychological burden of patients, and so as to stabilize the heart rate. Some studies have shown that the relaxation training of behavior and scientific comforting language can significantly reduce the impact of patients' bad emotions on their physical state, restore the homeostasis of internal environment, and successfully check.

In terms of heart rate control, the intervention group gave 25 mg Betaloc sublingual with a heart rate of more than 70 beats/min, with a maximum of no more than 100 mg. When necessary, oxygen inhalation was given to reduce the heart rate and stabilize the heart rate. The heart rate was controlled below 70 beats/min, which achieved good results and obtained the best image quality. In terms of breath control, good breath holding is a necessary and key factor for the successful completion of cardiac coronary artery examination. If the patient cannot hold his breath during the scanning process, the respiratory artifact is large, resulting in tomography and displacement of cardiac vascular image, which has a great impact on the image quality and has an impact on the diagnosis, which must be avoided [25].

## 5. Conclusion

In addition to the direct impact on heart rate and respiration, the quality of multislice spiral CT coronary imaging has a direct impact on its scanning technology, the amount of contrast medium, and the injection rate. Any improper operation may lead to the failure of the examination. Therefore, before apricot examination, giving patients careful and scientific nursing and controlling interference factors will help patients complete the examination better and faster and improve the image quality of coronary CTA. All patients in the intervention group obtained satisfactory images, which is inseparable from the careful nursing work before and during the examination. Careful nursing is an important guarantee for the success of the examination. To sum up, the nursing staff should fully communicate with the examinee before the contrast examination, and the appropriate combined application of metoprolol hydrochloride tablets can effectively control the examinee's tension, slow down the examinee's heart rate, and narrow the range of heart rate fluctuation during the examination. In addition, simple and easy breathing cooperation training can ensure better image quality, improve the success rate of examination and diagnosis accuracy, optimize the workflow, and give full play to the equipment and human resources. In a word, targeted nursing intervention can provide patients with high-quality, comprehensive, and scientific nursing service guidance. When used in patients undergoing coronary CT angiography, it can not only improve the examination quality but also reduce the artifacts caused by various influencing factors on the imaging image, meet the needs of diagnosis, promote the smooth progress of the examination, and improve the image quality.

## Figures and Tables

**Figure 1:** Coronary CT angiography.

**Figure 2:** Comparison of incidence and examination success rate of heart rate fluctuation amplitude > 10 BPM between the two groups.

**Table 1:** Excellent and good rate of comparative image quality (cases (%)).

Group	Number of cases	Excellent	Good	Poor
Observation group	50	42	8	0
Control group	60	31	12	7
*X* ^2^	—		7.623	
*P*	—		<0.05	

**Table 2:** Comparison of nursing effects.

Group	Number of cases	Inspection time	Nursing satisfaction
Observation group	50	5.54 ± 1.75	50
Control group	60	8.14 ± 1.34	41
*t*	—	7.356	9.836
*P*	—	<0.05	<0.05

**Table 3:** Comparison of basic heart rate and heart rate after health education between the two groups.

Group *n*	Basal heart rate	Heart rate after health education	*t*	*P*
Observation group 50	62.38 ± 3.58	94.26 ± 8.06	10.31	<0.001
Control group 60	63.49 ± 3.48	93.16 ± 6.23	8.87	<0.001
*t*	1.13	7.16		
*P*	>0.05	<0.001		

**Table 4:** Comparison of heart rate control time and breathing coordination training time between the two groups.

Group *n*	Heart rate control time (min)	Breathing coordination training time (min)
Observation group 50	52.37 ± 12.62	62.34 ± 11.24
Control group 60	31.63 ± 12.56	34.21 ± 6.37
*t*	6.91	10.35
*P*	<0.001	<0.001

## Data Availability

The data used to support the findings of this study are available from the corresponding author upon request.

## References

[1] Wang Y., Zhang D., Wei S. (2021). Effect of nursing intervention in the operating room based on simple virtual reality augmented technology on preventing gastrointestinal surgical incision infection. *Journal of Healthcare Engineering*.

[2] Yang J., Xu M., Wang Y., Gao Z. (2021). Analysis of the effect of intensive care based on lean nursing intervention. *Engineering*.

[3] Manal A. P., Fareed E., Elsayad H. (2021). Effect of selected nursing intervention on clinical outcomes among patients with nasogastric tube in intensive care units. *Japan Journal of Nursing Science*.

[4] Johnson A. K., Sherry Razo M. A. L., Smith J., Cain A., Detaranto B. (2021). A person centered nursing care intervention on a medical surgical unit. *Geriatric Nursing*.

[5] Liu H., Zhu D., Cao J., Jiao J., Wu X. (2019). The effects of a standardized nursing intervention model on immobile patients with stroke: a multicenter study in China. *European Journal of Cardiovascular Nursing*.

[6] Smeets C., Smalbrugge M., Koopmans R., Nelissen-Vrancken M., Zuidema S. U. (2020). Can the proper intervention reduce psychotropic drug prescription in nursing home residents with dementia? Results of a cluster-randomized controlled trial. *International Psychogeriatrics*.

[7] Faan A. B., Cauvin B. S., Msn A. C., Pretorius K., Johnson K. (2020). Application of project management tools and techniques to support nursing intervention research. *Nursing Outlook*.

[8] Yang J., Hu H., Li Y. (2020). Effect of dual-track interactive nursing intervention model on anxiety and depression in patients with coronary heart disease. *Psychiatria Danubina*.

[9] Msosa A., Bruce J., Crouch R. (2020). Effect of a formative assessment intervention on nursing skills laboratory learning in a resource-constrained country. *Nurse Education Today*.

[10] Zimansky M., Stasielowicz L., Franke I., Remmers H., Friedel H., Atzpodien J. (2020). Effects of implementing a brief family nursing intervention with hospitalized oncology patients and their families in Germany: a quasi-experimental study. *Journal of Family Nursing*.

[11] Sole M. L., Talbert S., Yan X. (2019). Nursing oral suction intervention to reduce aspiration and ventilator events (no-aspirate): a randomized clinical trial. *Journal of Advanced Nursing*.

[12] Alperovitch-Najenson D., Weiner C., Ribak J., Kalichman L. (2020). Sliding sheet use in nursing practice: an intervention study. *Workplace Health & Safety*.

[13] Spratling R., Faulkner M. S., Feinberg I., Hayat M. J. (2020). Creating opportunities for personal empowerment: symptom and technology management resources (cope-star) for caregivers of children who require medical technology. *Journal of Advanced Nursing*.

[14] Mcinnis L. A., Morehead A. (2020). Exercise as a therapeutic intervention. *Nursing Clinics of North America*.

[15] Kim H. S., Kang J. S. (2021). Effect of a group music intervention on cognitive function and mental health outcomes among nursing home residents: a randomized controlled pilot study. *Geriatric Nursing*.

[16] Brown L., Gardner G., Bonner A. (2019). A randomized controlled trial testing a decision support intervention for older patients with advanced kidney disease. *Journal of Advanced Nursing*.

[17] Baab C., Bakker A. C., de Vugt M. E. (2019). Effects of a Multidisciplinary Intervention on the Presence of Neuropsychiatric Symptoms and Psychotropic Drug Use in Nursing Home Residents WithYoung-Onset Dementia: Behavior and Evolution of Young-Onset Dementia Part 2 (BEYOND-II) Study. *The American Journal of Geriatric Psychiatry*.

[18] Cheung D., Tang S. K., Ho K., Jones C., Chiang V. (2021). Strategies to engage people with dementia and their informal caregivers in dyadic intervention: a scoping review. *Geriatric Nursing*.

[19] Williams K. A., Lee E. J., Wilmoth M., Selwyn C., Bydalek K. (2021). Screening, brief intervention, and referral to treatment/motivational interviewing school-based therapy pilot study. *Journal of Addictions Nursing*.

[20] Margaret B., George A., Phagdol T., Nayak B. S., Lewis L. E. (2022). Designing a mobile health intervention for preterm home care: application of conceptual framework. *Public Health Nursing*.

[21] Kofoed K. F., Engstrm T., Sigvardsen P. E., Linde J. J., Kber L. V. (2021). Prognostic value of coronary CT angiography in patients with non-ST-segment elevation acute coronary syndromes. *Journal of the American College of Cardiology*.

[22] Li G., Liu F., Sharma A. (2021). Research on the natural language recognition method based on cluster analysis using neural network. *Mathematical Problems in Engineering*.

[23] Xin L., Jianqi L., Jiayao C., Fangchuan Z. (2021). Mn_2_O_3_/*γ*-Al_2_O_3_ catalysts synergistic double dielectric barrier discharge (DDBD) degradation of toluene, ethyl-acetate and acetone. *Chemosphere*.

[24] Huang R., Yan P., Yang X. (2021). Knowledge map visualization of technology hotspots and development trends in China’s textile manufacturing industry. *IET Collaborative Intelligent Manufacturing*.

[25] Jayakumar J., Nagaraj B., Chacko S., Ajay P. (2021). Conceptual implementation of artificial intelligent based E-mobility controller in smart city environment. *Wireless Communications and Mobile Computing*.

